RETRACTED

# EST–SSR Marker Development and Full-Length Transcriptome Sequence Analysis of Tiger Lily (*Lilium lancifolium Thunb*)

**DOI:** 10.1155/2022/7641048

**Published:** 2022-01-28

**Authors:** Mingwei Sun, Yilian Zhao, Xiaobin Shao, Jintao Ge, Xueyan Tang, Pengbo Zhu, Jiangying Wang, Tongli Zhao

**Affiliations:** ^1^Lianyungang Academy of Agricultural Sciences, Lianyungang, China; ^2^Nanjing Forest University, Nanjing, China

## Abstract

The fast advancement and deployment of sequencing technologies after the Human Genome Project have greatly increased our knowledge of the eukaryotic genome sequences. However, due to technological concerns, high-quality genomic data has been confined to a few key organisms. Moreover, our understanding of which portions of genomes make up genes and which transcript isoforms synthesize these genes is scarce. Therefore, the current study has been designed to explore the reliability of the tiger lily (*Lilium lancifolium Thunb*) transcriptome. The PacBio-SMRT was used for attaining the complete transcriptomic profile. We obtained a total of 815,624 CCS (Circular Consensus Sequence) reads with an average length of 1295 bp. The tiger lily transcriptome has been sequenced for the first time using third-generation long-read technology. Furthermore, unigenes (38,707), lncRNAs (6852), and TF members (768) were determined based on the transcriptome data, followed by evaluating SSRs (3319). It has also been revealed that 105 out of 128 primer pairs effectively amplified PCR products. Around 15,608 transcripts were allocated to 25 distinct KOG Clusters, and 10,706 unigenes were grouped into 52 functional categories in the annotated transcripts. Until now, no tiger lily lncRNAs have been discovered. Results of this study may serve as an extensive set of reference transcripts and help us learn more about the transcriptomes of tiger lilies and pave the path for further research.

## 1. Introduction

The tiger lily (*Lilium lancifolium Thunb*) grows from bulbs producing corolla-shaped flowers of various colors, such as orange, red, yellow, and white [1]. The tiger lily is well-known across the globe for its beautiful look as well as is used as a nutritious food. In addition, the Chinese Ministry of Health's medical plants listed tiger lily as a medicinal plant because of its abundant minerals and bioactive constituents including alkaloids, phenolic glycosides, pectin, and vitamins. The tiger lily has a large genome, ranging from 32.8 to 47.9 pg [2], as a triploid plant. Full-length sequencing has a lot of promise for transcriptomic evaluation since it serves as a convenient and cost-effective approach to annotate nonmodel species' transcriptomes [3]. The full genomic and transcriptomic data would be extremely useful for studying the gene models of the tiger lily. However, the enormous and unidentified genome, as well as the high heterozygosity, makes the functional evaluation of genes challenging.

RETRACTED

In transcriptome studies, the next-generation sequencing (NGS) platform provides active transcriptional patterns and has obtained considerable scientific interests in the last ten years [4]. Given the fact that gene expression can be precisely analyzed with high throughput resequencing, some significant transcriptional data covering long lengths, such as simple sequence repeats (SSRs), alternative-splicing (AS), and long noncoding RNA (lncRNA), might be lost because RNA or cDNA must be segmented while preparing the sample and only short-read data can be accessed with NGS platforms. Long-read sequencing technologies capable of providing complete cDNA molecules, such as Oxford Nanopore Technologies (ONT) and Pacific Biosciences (PacBio), are available to meet the study requirement [5, 6]. Due to the ability of PacBio to obtain the complete length of transcripts, gene annotation, isoform, and lncRNA detection, precision has been significantly improved relative to the NGS systems [7, 8]. The long-read sequencing technologies are powered by the PacBio-SMRT sequencing approach. Long readings and great accuracy are provided by SMRT sequencing. As a result, PacBio-SMRT isoform sequencing (Iso-Seq) has been utilized in numerous animals and plants for transcriptomic profiling [9, 10].

Only histological and transcriptomic analysis of *Lilium ancifolium* during bulbil formation has been carried out [11]. Moreover, SMRT and Illumina-based seq have been carried out in certain plants (X. Y. [12, 13]). Until now, no tiger lily lncRNAs have been discovered. In the current research work, the PacBio-SMRT approach has been used to sequence the entire cDNA library of tiger lily. The RNA-seq from the Illumina HiSeq plant was combined, and the full-length transcriptomes (FLTs) were obtained in order to identify and quantify the isoform transcripts. This dataset could serve as a source of rich data regarding full-length cDNA sequences, which could help us learn more about the tiger lily. The functional annotation of the underlined FLTs, as well as the discovery of lncRNAs, will aid our understanding of gene functions. Herein, we have designed the SSR primers which could play an important role in the tiger lily's breeding, affinity, and gene mapping as well as its systematic classification. As a result of these findings, effective methods for gene research and breeding could be developed.

## 2. Materials and Methods

### 2.1. Collection of Plant Samples

The Lianyungang Academy of Agricultural Sciences (China) grew the tiger lily (*Lilium lancifolium Thunb*). After growing, the scale samples were collected from three different tiger lily plants. The samples were then frozen with liquid nitrogen, followed by keeping them at -70°C and storing till further use.

RETRACTED

### 2.2. PacBio ISO-Seq

The Iso-Seq library was created via Pacific Biosciences' Iso-Seq technique with the Clontech-SMARTer-PCR-cDNA-Synthesis-Kit and the BluePippin Size Selection System procedure (PN 100-092-800-03). The obtained data was uploaded to the Sequence Read Archive (SRA) (accession no. #SRR8903502) of the NCBI server.

### 2.3. PacBio ISO-Seq Analysis

The SMRTlink-version-7.0 (https://www.pacb.com/support/software-downloads/) was employed to process the raw readings, followed by generating a Circular Consensus Sequence (CCS). Based on whether a poly-A tail, 5′, or 3′ primer was present, the CCSs were separated into reads as full-length or non-full-length. We designed the ICE (Iterative Clustering for Error-Correction) algorithm for the prediction of consensus isoforms from FLTs (full-length transcripts), while quiver version 1.1.0 (California, USA) was employed to polish the consensus isoforms with non-FLTs [14]. Those sequences containing no repetition or extension on either end were considered transcripts. PacBio readings were aligned with Illumina RNA-seq data using the tool LoRDEC to validate sequence accuracy [15]. The ultimate consensus isoforms for the ensuing study were collected after CD-HIT (W. [16]) and eliminated all redundancies in the corrected consensus reads.

### 2.4. Annotation of the Transcriptome

The isoforms were analyzed using databases, i.e., KEGG, nonredundant (NR) protein sequences [17], Clusters of Orthologous Groups of proteins (COGs) [18], and Swiss-Prot [19] with NCBI-blast (version-2.7.1) and diamond (version-0.8.36) (*E*‐value ≤ 1 × 10^−5^) [20]. The Pfam analysis and GO term annotations [21] were performed using HMMER (version 3.1) [22] and Blast2GO (version 2.5.0) [23], respectively.

### 2.5. Detection of CDS, TF, lncRNA, and SSR

Simple sequence repeat (SSR), transcription factor (TF), and coding DNA sequence (CDC) were assessed using MISA [24], iTAK [25], and ANGLE [26] software. The lncRNAs were retrieved followed by employing CNCI [27], CPC2 [28], Pfam [21], and PLEK (https://sourceforge.net/projects/plek/) to evaluate each transcript with the ability to code. For SSR recognition, MISA-version 1.0 [24] was used. The parameters were specified for identifying mononucleotide to hexanucleotide unit sizes having a minimum repetition of 10, 6, 5, 5, 5, and 5, accordingly. Batch Primer-3 was employed to design SSR primers. To confirm the SSR primers' applicability [29], the DNA template of tiger lily was amplified by PCR, followed by separating the PCR product by using polyacrylamide gels (8%).

RETRACTED

## 3. Results

### 3.1. The Isolation of FLTs from the Tiger Lily's Sepal

The RNA obtained from 5 plant samples was combined and sequenced on a PacBio Sequel system in order to acquire FLT data. Two SMRT cells retrieved 54.86 G subread bases from the PacBio library, giving 815,624 CCS reads with an average length of 1295 bp, as shown in Table 1. Full-length reads with the 5′ primer, 3′ primer, and poly-A tail accounted for 461,744 (56.62%) of the total reads, while FLNC (full-length reads nonchimeric) sequences accounted for 459,322 (56.32%), as represented in Table 1. We generated 38,707 polished consensus FLTs (average length of 1574 bp) using the ICE Quiver and Arrow polishing algorithms (Table 1). FLNC sequences were adjusted with Illumina short-read RNA-seq reads using LoRDEC in order to increase consensus accuracy. Consequently, in 38,707 transcripts, 8596 nucleotides were found to be revised, although the average length remained at 1574 bp, as shown in Table 1. The majority of transcripts (98.3%) have sequence lengths ranging from 0.2 to 4 kb (Figure 1). The repetitive and identical sequences for one unigene were eliminated using the software CD-HIT. A total of 15,608 unigenes with an average length of 1627 base pairs were retrieved using the CD-HIT software (with a 95% cutoff point) (Figure 1 and Table 2).

### 3.2. Prediction of Transcription Factor

Transcription factors, as the master regulators of gene expression, are critical for plant growth and resistance to biotic as well as abiotic stressors. Herein, 768 TFs were discovered and grouped into 30 families. Around 64, 47, 44, 42, 42, 42, 41, 40, 40, 37, and 32 Te TFs (in the tiger lily transcriptome) associated with MADS-MIKC, MADS-M-type, MYB-related, C3H, FAR1, bZIP, C2H2, GRAS, bHLH, AP2/ERF-ERF, and MYB families with 8.33%, 56.12%, 5.73%, 5.47%, 5.47%, 5.47%, 5.34%, 5.21%, 5.21%, 4.82%, and 4.17% abundance, accordingly (Figure 2). The TFs' gene sequence character would be quite helpful in gene functional analyses and would be a great starting point for quick gene discovery.

### 3.3. Simple Sequence Repeat (SSR) Analysis

SSR markers are critical in the construction of DNA fingerprinting, high-density genetic maps, and phylogenetic evolutionary studies due to their codominance, stability, high repeatability, primer specificity, high polymorphism, and ease of detection. Around 3319 SSRs were discovered in 2968 unigenes during this study. There were 2675 transcripts with a single SSR locus and 293 transcripts with two or more SSR loci. The most prevalent motif type was composed of mono- (1039), di- (862), and tri- (766) repeats (Figure 2). Primers (128 pairs) were designed based on the SSR primer information for successful amplification of the cDNA, but only 105 (82.03%) primer pairs were able to generate PCR products using whole genomic DNA as the template.

RETRACTED

### 3.4. Identification of lncRNA

lncRNAs are a class of noncoding poly-A RNAs that regulate gene expression via altering dosage compensation, as well as epigenetic and cell-cycle regulation. lncRNAs were identified using four different computational approaches, including the CNCI, Pfam (Protein Family), PLEK, and CPC databases. These four approaches were combined to produce comprehensive lncRNA data. A total of 824, 3147, 5457, and 1962 lncRNAs were evaluated using the databases CNCI, Pfam, PLEK, and CPC, accordingly (Figure 3). Only 570 in 6852 lncRNAs were found to be shared across the four databases, as shown in Figure 3.

### 3.5. Functional Annotation of Transcripts

NR protein sequences, Swiss-Prot, KEGG, KOG, GO, NT (NCBI nucleotide sequences), and Pfam databases were used to functionally assess and classify the unigene sequences. Around 14,614, 12,575, 14,554, 9650, 10,705, 11,309, and 10,705 were detected and annotated in the NR, Swiss-Prot, KEGG, KOG, GO, NT, and Pfam databases, accordingly, as depicted in Figures 4 and 5. The underlined databases shared 6656 unigenes in common. Elaeis guineensis has the highest percentage of unigenes (32.65%), according to the species distribution annotation. Following that, *Phoenix dactylifera*, *Musa acuminata*, *Ananas comosus*, *Asparagus officinalis*, Nelumbo nucifera, *Anthurium amnicola*, *Vitis vinifera*, and *Lilium longiflorum* had a high proportion of unigenes, with the percentage of 25.82%, 8.11%, 7.15%, 5.29%, 2.30%, 2.20%, 0.79%, and 0.72%, accordingly, as indicated in Figure 6.

### 3.6. GO Analysis

To further identify the gene functions, GO analysis of the unigenes was performed. According to GO enrichment, 10,706 unigenes were classified into 52 functional groupings, which were separated into three classes: biological process (BP), cellular component (CC), and molecular function (MF). In the BP, 5188, 4676, and 3044 unigenes contributed in metabolic cascades, cellular processes, and single-organism processes, accordingly. In the CC, 2258, 2258, 1594, 1282, and 1136 unigenes were found to be associated with the cell, part of the cell, cellular organelle, complex containing macromolecules, and membrane, accordingly. In the MF group, 6393, 4851, and 473 unigenes were involved in interacting and binding activities, catalysis, and transportation, accordingly, as indicated in Figure 7.

RETRACTED

### 3.7. KEGG Classification

Unigenes (14554) were mapped to KEGG functional pathways (354), and the pathways were subsequently categorized into different groups, as shown in Table 2. Functional analysis revealed that unigenes were mostly enriched in the ribosome (434) and metabolic pathways including carbon metabolism (345), as represented in Table 2. This classification offered useful information for finding specific tiger lily processes, functions, and pathways.

### 3.8. KOG Classification

Each unigene was evaluated with the Clusters of KOG database to investigate the functional annotation and characterization of the tiger lily unigenes. The results suggested that 9650 unigenes could be categorized into 25 different groups which have been represented in the form of alphabets, as shown in Figure 8. The highest category among these was general function prediction, which had the most unigenes (1709, 15.88%). Moreover, defense mechanisms, ECM, cellular migration, and nuclear components had percentages of less than 1%, as shown in Figure 8.

## 4. Discussion

Obtaining genomic data is essential for comprehending and expanding the study of a species. In comparison to whole-genome sequencing, transcriptome sequencing is less expensive and more suited to studying the genomes of multiple plant species [30]. Third-generation FLT sequencing relies on PacBio-SMRT sequencing and has the benefit of a long read-length and good precision over standard second-generation sequencing methods. As an effective and accurate approach for screening FLTs, and SMRT sequencing has been crucial in advancing the field of complete transcriptomic profiling, particularly for those plants lacking the reference assembly. Without any of the requirements for assembling, the underlined approach could provide single-molecule full-length mRNA information and reliably highlight areas including gene families, AS, and lncRNA.

As a rapid and relatively convenient approach for screening FLTs, SMRT sequencing technology has greatly contributed to whole-transcriptome profiling research, specifically for those plants lacking the reference assembly. In the current study, the SMRT sequencing tools (based on the PacBio Sequel platform) were used to sequence the whole transcriptome of the tiger lily. A total of 63.85 Gb of sequencing data, comprising 815,624 CCS and 459,322 FLNC reads, were generated to ensure sequencing accuracy. FLNC reads made up 56.31 percent of all CCS reads, which is similar to the results in alfalfa and strawberry [31](Y. [32]). While next-generation sequencing systems could precisely quantify gene expression, large nucleotide sequences were frequently missed. Transcripts obtained using SMRT sequencing approaches are typically longer than those obtained using next-generation sequencing technologies, where one read indicates an FLT [33]. According to our obtained results of SMRT sequencing, tiger lily's average length of transcripts comprised of 72,076 bp which is significantly longer than the lengths attained previously using Illumina sequencing (114.59 bp-297.76 bp) ([12, 13]). Additionally, we discovered that 97.45 percent of all transcripts in this SMRT sequencing result were longer than 2000 bp, demonstrating that PacBio's SMRT sequencing approach is an efficient and effective method for investigating transcript sequence information, particularly for long transcript sequences.

RETRACTED

TFs are types of regulatory factor that influences gene expression. TFs are associated with the regulation of fine-tuning gene expression in cellular differentiation, development, and several other activities of cells, notably against abiotic stress and plant diseases, by combining lncRNA, microRNA, and methylation [34, 35][36]. The regulatory network in plants has been the subject of an increasing number of studies in recent years. Until now, no tiger lily lncRNAs have been discovered. The tiger lily transcripts yielded 768 transcription factors and 6852 lncRNAs, which will be beneficial for future tiger lily research.

SSR primers are a good approach to map genes and analyze genetic variation and gene function, both of which are crucial for breeding purposes because the tiger lily genome has not yet been examined. It was easy to construct high-quality SSR makers because of the extensive transcript sequence data. According to the polished gene sequences, a total of 3319 SSRs were found in 2968 unigenes. SSR repeat motifs ranging from 1 to 6 nucleotides account for approximately 41.32% of the 6 types of repeat motifs, with di- and trinucleotide motifs accounting for the rest. A/T, AT/AT, and CCG/CGG were the most common mono-, di-, and trinucleotide motifs in this analysis. The most common nucleotide repeat motif is A/T, which accounts for around 39.59% of all nucleotide motifs and is considered to be abundant in plant genomic sequences [37], and AT/AT and AG/CT, which belong to the dinucleotide motifs, account for 15.94% and 14.41%, respectively. CCG/CGG is the most common trinucleotide motif, accounting for 9.01% of all motifs, followed by AGG/CCT and AGC/CTG with the percentages of 3.93% and 3.65%, accordingly. Moreover, 128 pairs of primers were created to assess the reliability of makers based on the knowledge regarding the SSR marker. Following that, the underlined primers were able to successfully amplify PCR products when the cDNA was utilized as the template for PCR amplification. However, when whole-genomic DNA was utilized as a template, only 105 primer pairs (82.03%) effectively produced PCR products. The lengthy intron in the targeted area and the primer nucleotide's location on two adjoining exons may have contributed to the failure of PCR amplification of 23 pairs of primers previously described. The highlighted findings suggest that the created SSR markers based on the PacBio-SMRT sequencing approach contribute significantly to genetic investigations (in tiger lily) and could be useful in tiger lily breeding research.

RETRACTED

## 5. Conclusion

Herein, we analyzed the tiger lily's FLTs through PacBio's SMRT sequencing technology. This is the first time the tiger lily's transcriptome has been sequenced using third-generation long-read technology. Results of the acquired transcriptome data showed 38,707 unigenes, 6852 lncRNAs, and 768 TFs in tiger lily. According to our obtained results of SMRT sequencing, tiger lily's average length of transcripts comprised of 72,076 bp which is significantly longer than the lengths obtained previously using Illumina sequencing. Moreover, 3319 SSRs were identified, and 105 out of 128 primer pairs significantly amplified PCR products. The transcriptomic data and SSR markers generated in this study may ease future genetic investigations, aid in the breeding of novel tiger lily variants, and pave the path for further research.

## Figures and Tables

**Figure 1:** The transcript (38,707) and unigene (15,608) length distribution in tiger lily sepals.

**Figure 2:** Transcript families and their corresponding numbers of TFs in the tiger lily.

**Figure 3:** Prediction of lncRNAs using CNCI, CPC, CPAT, and Pfam analysis tools, as indicated in the Venn diagram.

**Figure 4:** Frequency and distribution of SSRs on the basis of the motif.

**Figure 5:** Venn maps of the unigenes among NR, GO, KEGG, Pfam, KOG, NT, and Swiss-Prot databases.

**Figure 6:** Homologous species distribution of tiger lily transcripts annotated in the NR database.

**Figure 7:** GO classification of tiger lily transcripts. BP, CC, and MFs are indicated by red, green, and blue colors, accordingly.

**Figure 8:** The KOG classification of tiger lily transcripts. The *x*-axis and *y*-axis represent the subcategories and the number of transcripts, accordingly.

**Table 1:** Representation of Iso-Seq from the sepal of *Lilium davidii* var. unicolor Salisb by PacBio Sequel system.

SMRT cells	Subread base (G)	Reads of CCS	Non-full-length reads	Full-length reads	FLNC reads	Consensus transcripts	Mean length (bp)	Unigenes
	54.86	815,624	353,880	461,744	459,322	38,707	1574	38,707

RETRACTED

**Table 2:** Summary of the unigenes mapped to KEGG functional pathways.

Number	Pathway ID	Pathway name	Unigene number
1	ko03010	Genetic information processing, translation, ribosome	434
2	ko01200	Metabolism, global and overview maps, carbon metabolism	345
3	ko01230	Metabolism, global and overview maps, biosynthesis of amino acids	307
4	ko04141	Genetic information processing; folding, sorting, and degradation; protein processing in the endoplasmic reticulum	253
5	ko03040	Genetic information processing, transcription, spliceosome	236
6	ko00190	Metabolism, energy metabolism, oxidative phosphorylation	207
7	ko05169	Human diseases; infectious diseases: viral; Epstein-Barr virus infection	180
8	ko04144	Cellular processes, transport and catabolism, endocytosis	179
9	ko00010	Metabolism, carbohydrate metabolism, glycolysis/gluconeogenesis	175
10	ko03013	Genetic information processing, translation, RNA transport	166
11	ko05016	Human diseases, neurodegenerative diseases, Huntington's disease	161
12	ko00230	Metabolism, nucleotide metabolism, purine metabolism	156
13	ko04075	Environmental information processing, signal transduction, plant hormone signal transduction	152
14	ko00620	Metabolism, carbohydrate metabolism, pyruvate metabolism	146
15	ko05418	Human diseases, cardiovascular diseases, fluid shear stress and atherosclerosis	135

## Data Availability

The corresponding author can provide information about this work upon reasonable request.
